# The Psychological Education Strategy of Music Generation and Creation by Generative Confrontation Network under Deep Learning

This article has been retracted.

**DOI:** 10.1155/2022/3847415

**Published:** 2022-06-13

**Authors:** Jiaxin Hu, Zhaohui Ge, Xiaohua Wang

**Affiliations:** ^1^School of Music and Dance, Qiqihar University, Qiqihar, China; ^2^College of Preschool Education, Xiangzhong Normal College for Preschool Education, Shaoyang 422001, China; ^3^College of Music, Qinghai Normal University, Xining 810016, China

## Abstract

In order to study the role of generative adversarial network (GAN) in music generation, this article creates a convolutional GAN-based Midinet as a baseline model through the music generation process and creative psychological education and GAN principle. Additionally, it proposes a music generation model based on music theory rules and a chord-constrained GAN dual-track music generation model. Based on this model, a deep chord gated recurrent neural generative adversarial network (DCG_GAN) is proposed. The generated melodies are evaluated in both subjective and objective directions. The results show that the three evaluation indicators of DCG_GAN have the highest scores in the subjective evaluation. The average score given by ordinary listeners reaches 3.76 points, and the professional score reaches 3.58 points, which are 0.69 and 1.31 points higher than the baseline model, respectively. In the objective evaluation, DCG_GAN is improved by 8.075% in empty bars rate (EBR). The UPC (num_chroma_used) evaluation index value of the DCG_GAN model is improved by 0.52 compared with the baseline model. The qualified note ratio (QNR) evaluation index value is improved by up to 4.46% among the five audio tracks. The proposed overall style-based music generation model has superior performance in music generation. Both subjective and objective evaluations show that the generated music is more favored by the audience, indicating that the combination of deep learning and GAN has a great effect on music generation.

## 1. Introduction

With the development of computer technology, the application of deep learning technology in the direction of music generation provides a new creative mode for music creation. Deep learning is a field of machine learning inspired by neural architecture. These networks automatically extract features from data sets and can learn any nonlinear function. Shen et al. [1] pointed out that the media has changed the way people communicate with friends. Generative adversarial networks (GANs), as the state-of-the-art method for generating high-quality images, also show unique advantages in the direction of music generation [2]. Automatic music generation is the process of creating a short piece of music with minimal human intervention, and algorithmic composition enables machines to create music. This makes music creation no longer only for professional composers, and music lovers can also create their favorite melodies through machine creation [3]. The combination of artificial intelligence and intelligent manufacturing has laid the foundation for the generation of intelligent musical instruments, which can not only expand the types of musical instruments but also apply intelligent musical instruments in music education. The combination of intelligent technology and hardware and software makes complex playing skills easier to learn and boring training process into fun.

In addition to traditional tasks such as prediction, classification, and translation, deep learning as a method of music generation has also received increasing attention for direct application. Deep learning to generate content quickly reaches its limits, generating content that tends to mimic the training set without showing true creativity. Furthermore, deep learning architectures do not provide a direct method of control generation [4]. Conditional distributions generated by the joint probabilities of all pixels or words achieve state-of-the-art results in content generation tasks by means of neural network methods in deep learning. These models accomplish their tasks by modeling many random variables. Starting from Mozart's random algorithm to determine musical scores by rolling dice and the rule-based vowel-pitch algorithm designed by Guido darezo, human exploration of automatic music generation algorithms has never stopped. In the deep learning era, the massive increase in computing power enables us to implement more complex algorithms. One of the mainstream approaches in machine learning algorithms is based on neural networks. The task of controlled music generation has been plagued by the central question of how much control and constraints humans should impose on the model. If humans apply too many inductive biases and rules to control the basic logic of music generation, then music generation models will be uncreative; if humans only impose weak constraints on the model, the music generated by the model is often not usable by humans.

The methods of literature research and model building are adopted. Through the research of different music generation methods, a convolutional GAN model based on chord constraints is innovatively proposed based on deep learning. The music generation based on the overall style can make up for the problem of the lack of music types and easy repetition in the current music generation technology. The model is adopted to generate more pleasing, rhythmic, and diverse music eventually, and the same conclusion is reached through both subjective ratings and objective evaluations by listeners. The research framework consists of four parts.  Section 1 is the introduction and literature review to introduce the research background and research significance, as well as recent research work in related fields.  Section 2 is the research method through the psychology of music generation and creation. The research of GAN proposes a music generation model based on chord constraints and overall style and conducts experimental verification.  Section 3 results illustrate the data results and analysis of the validated model proposed in the Methods section.  Section 4 concludes with a summary of the current study and points out the limitations and prospects of the study.

## 2. Literature Review

Music has a rich representation. Any musical abstraction can be viewed as a representation of music. For example, in the music labeling task, as the model labels the music, the model also learns to extract representations from the music. Briot [5] provided a music generation tutorial based on deep learning techniques. After a brief introduction to the subject illustrated by a recent example, some early works of music generation using artificial neural networks foreshadowed current technology. Dua et al. [6] leveraged deep learning techniques such as recursive neural networks (RNNs) with gated recurrent unit (GRU) and long-short-term memory (LSTM) in the source separation module, the multi-layer GRU used to implement the RNN in the chord estimation module, the LSTM unit was used to implement the RNN. In the source separation module, the number of sources that can be separated is also increased to improve the accuracy of the chord estimation module. Goienetxea et al. [7] proposed to use the melody coherence structure extracted from template fragments to generate coherent melody, which was applied to generate bertso melody, and added the generation of melody rhythm content, for which the rhythm of template fragments was also created coherent structure. Lopez Duarte [8] addressed excessive repetition caused by low interactivity of musical sequences during gameplay by using random or sequential containers with overlapping rules and adaptive mixing parameters. Li and Sung [9] proposed a conditional GAN method using an initial model. This method can automatically generate complete variable-length music.

To sum up, most of the current neural network models for music generation are RNNs or their derivatives. The music generated in this way often uses preset music information as the generating premise of the current music segment, which limits the types of music generation to a certain extent and is easy to repeat. However, when a single neural network uses GAN to generate music, it is prone to mode collapse and unstable performance. It is necessary to develop a new deep neural network model for music creation.

## 3. Materials and Methods

### 3.1. Music Generation and Creation Psychology

Using the music generation of AI can capture the characteristics of real music by computer, and music creation can be carried out independently [10]. The psychological structure of the main body of music creation consists of the composer's inherent physiological quality, environmental education, training, and external stimulation, which interact in the process of practice and gradually develop [10]. Shen et al. [11] applied a text mining method called double-layer concept link analysis, which is a combination of many psychological factors, such as perception, memory, thinking, imagination, and aesthetic experience. In the process of creation, these numerous psychological factors do not appear in an orderly way but are characterized by integrity, organization, and variability, often between various complex psychological factors and technologies, and finally achieve a balance [12].

In multi-track music generation, the commonly used music structured symbols are represented as musical instrument digital interface (MIDI) [13]. As a communication standard between musical instruments and computers, MIDI has been widely used since it was proposed, which is a protocol for recording the connection mode and information between musical instruments and computers [14]. Compared with other text formats, MIDI contains more information and can be used to assist in music creation. It has been named “music score that can be understood by computer” by the composition industry [15]. The basic idea of MIDI is to use note control signals to make music. Now, most music is created by combining MIDI and various timbres in the timbre library [16].  Figure 1 indicates the parsing process of MIDI files.

In Figure 1, a schematic diagram of the process of parsing a MIDI file is shown. Firstly, a MIDI file analyzer is used. The note information and auxiliary information in the file are analyzed. Then, the integration analyzer integrates the note information recorded in the MIDI file according to some auxiliary information to obtain the staff. MIDI files have 16 channels, and up to 16 instruments can work simultaneously. There is no one-to-one correspondence between tracks and channels, and there can be many correspondences. The performances of different parts are placed in different tracks without interfering with each other. As a form of visual music storage, the Piano roll [17] is represented by a set of coordinate axes, time, and pitch and has been widely used as the storage of visual music data. But Piano Roll has now been replaced by the MIDI file format. MIDI representation represents a new way of storing musical performance data. It performs the mechanical operation of the piano roll format both digitally and electronically [18]. However, many software for processing music performance files stored in MIDI data often uses Piano Roll representation to display and analyze the characteristic information of music [19].

### 3.2. GAN Model

GAN has two networks: a generator and a discriminator. The two networks can be different neural networks. The data set used in the training of the music generation model based on convolutional GAN is the preprocessed melody bars of popular music melodies in the .npz format. Hyperparameter setting: the number of bars is 50496 bars (bar), the size is 789 MB, the number of chord bars is 50496 bars, the memory size is 5.01 MB, the dimension is 13 dimensions, the format is piano roll format, a data set with 16 note units, a pitch range of C4–B5, and a random noise with a length of 100 Gaussian white noise.

The music generation process is used to illustrate how GAN work, as shown in Figure 2.

In Figure 2, there are two networks in the structure of GAN, namely the generator network Generator (*G*) and the discriminator network Discriminator (*D*). GAN mainly trains the neural generator network and the discriminator neural network to make the two networks play a game and finally obtain better results for the two networks. Suppose *G* is a generation network for a piece of music, input a random noise *z*, and generate music fragments through it, denoted as *G*(z). *D* is a music identification network that is used to confirm whether this piece of musical material is “real.” Its input parameter is *x*, which represents a piece of music. The output *D*(*x*) represents the probability that *x* is real music. If it is 1, 100% is real music. Otherwise, the output is 0, which is not real music at all.

In the training process, the generation network *G* tries to generate real music clips to deceive the identification network *D*, and the identification network *D* tries to distinguish the music generated by *G* from the real music. In this way, *G* and *D* constitute a dynamic “gaming process.” Finally, as a result of the game, *G* can generate enough music *G*(*z*) to “confuse the false with the true.” For *D*, it is difficult to determine whether the music generated by *G* is real, so *D*(*G*(*z*)) = 0.5. The following equation demonstrates the objective function to be optimized in this process.

(1) $$\begin{array}{c} \underset{G}{\min}\underset{D}{\max}V\left(G,D\right)=\underset{G}{\min}\underset{D}{\max}\left[E_{p_{\text{data}}\left(x\right)}\left[\text{log}D\left(x\right)\right]+E_{p_{z}\left(z\right)}\left[\text{log}\left(1-D\left(G\left(z\right)\right)\right)\right]\right], \end{array}$$

where *p*_data_(*x*) means the probability distribution of real data defined in the data space *x*, *p*_*z*_(*z*) represents the probability distribution *z* of potential variables defined in the potential data space *z*. *V*(*G*, *D*) is a binary cross-entropy function, usually used in the binary classification problems. From the perspective of *D*, if the sample comes from real data, *D* will maximize its output; If the sample is from *G*, *D* will minimize its output. Meanwhile, *G* wants to deceive *D*, so when false samples are presented to *D*, it tries to maximize the output of *D*. The optimal discriminator can be solved out by deriving *V*(*G*, *D*).

(2) $$\begin{array}{c} D^{*}\left(x\right)=\frac{p_{g}\left(x\right)}{p_{g}\left(x\right)+p_{\text{data}}\left(x\right)}. \end{array}$$

The generation of the confrontation network is the process of the game through *G* and *D* neural networks, which finally makes the two networks reach the optimal state. It generates a fake music generator and a high-level music discriminator [20–22]. The input music may be fake music or real music, which is identified by the discriminator. If it is real music, the output result is true. If it is fake music, the judgment result is false. Additionally, feedback is given to the generator to improve its generator performance. In this cycle, finally, a generator is formed, which can generate highly similar music, and a high-level music discriminator is also formed [23].

### 3.3. Music Generation Model Based on Convolutional GAN

Midinet (a convolutional GAN for symbolic-domain music generation) [24–26] is used as the baseline model to apply the convolutional GAN to the field of music generation, which is composed of regulator, generator, and discriminator CNN.  Figure 3 indicates the structure of the model.

In Figure 3, the two-dimensional start-up subsection is used as input through four convolutional layers, and the output is combined with each layer of CNN of the generator. One-dimensional chords and random noise are input into the generator together. After four layers of convolutional layers, they are combined with the starting bars generated by the regulator to generate new melodies. In the discriminator, the input is the real melody or the generated melody, and the starting bar and chord are added. The discriminant result is output through two layers of convolution and one layer of full connection.

The following equation refers to the overall objective equation of the model:

(3) $$\begin{array}{c} {\text{minmax}}_{G}V\left(G,D\right)=\left[E_{x∼p_{\text{data}}\left(x\right)}\left[\text{log}D\left(x\right)\right]+E_{z∼p_{z}\left(z\right)}\left[\log\left(1-D\left(G\left(z\right)\right)\right)\right]\right]. \end{array}$$

Calculation of the discriminator CNN accords to the following equation:

(4) $$\begin{array}{c} \underset{D}{\text{max}}\left[E_{p_{\text{data}}\left(x\right)}\left[\text{log}D\left(x\right)\right]+E_{p_{z}\left(z\right)}\left[\log\left(1-D\left(G\left(z\right)\right)\right)\right]\right]. \end{array}$$

The calculation of generator CNN is as follows:

(5) $$\begin{array}{c} \underset{G}{\min}E_{x_{N}p\left(x\right)}\left[\text{log}\left(1-D\left(G\left(z\right)\right)\right)\right]. \end{array}$$

In equations (3)–(5), *x* ~ *p*_data_(*x*) represents sampling from real data, *z* ~ *p*_*z*_(*z*) represents sampling from random distribution, *D* represents the discriminator network, and *G* represents the generator network. *D*(*x*) represents the data of the discriminator network and *D*(*G*(*z*)) represents the probability that the generator in the discriminator network runs out of noise. The data *x* results from the generated data, the Gaussian noise *z*. The discriminator and generator network structures are shown in Figure 4:

In Figure 4(a), if the data come from real data, the discriminator probability is the maximum value. The purpose of log transformation is like log-likelihood, which does not affect the monotonicity of the function, but makes the operation simpler. If the data come from a Gaussian noise distribution and the input to the discriminator is the result generated by the generator, then the probability of the discriminator network drops. In Figure 4(b), the data *x* come from the generated data, that is, the result of Gaussian noise *z*, then the probability of *D*(*G*(*z*)) will rise, and the probability of log(1 − *D*(*G*(*z*)) will drop, and finally the minimum value of the generator network is obtained.

### 3.4. Dual-Track Music Generation Model of GAN Based on Chord Constraint

#### 3.4.1. Music Generation Data Set and Compilation Environment

The music generation data set adopts the PyTorch network framework [27] to generate the data set used for melody. The data format is MIDI. Besides, a dual track of melody and chord is adopted, and the number of melody bars is set to 50496 bars. Initially, the data set needs to be preprocessed.  Figure 5 demonstrates the process of preprocessing.

In Figure 5, when the data set is preprocessed, the note unit must be fixed first, and the melody is set to *w*=16. Then, some short notes, triplets, and data whose starting notes are a rest need to be deleted, and the pitch converted. The 128 notes in piano roll format are converted to two octaves *C*4 − *B*5, ignoring velocity. The MIDI format is adopted for representation, and then the twelve equal-tempered keys are cycled to output the final data set.

*X*(*h∗w*) represents the input melody, *h* denotes the note data in MIDI format, and *w* refers to the time step of a section. Representation form adopts sparse matrix form and is composed of one-hot coding, *X* ∈ {0,1}*h∗w*. There are 128 pitch states, so (1128) is used to represent each note. The effective pitch table is 1 and other registers are 0. The size of melody bars is 789 MB, the number is 50496, and the actual pitch is 24. Chord bars are 13 dimensions, 50496 in number, and 5.01 MB in size. The first twelve dimensions represent the range of pitch, and the last one represents the label of major or minor. The data set contains three parts: real melody, start section, and chord. The real melody and start section of the data set are allocated to the training set and test set according to 9 : 1.

The model editing environment settings are shown in Table 1:

#### 3.4.2. Music Generation Model Based on Music Theory Rules

In Midinet, fixed chords are used for music generation, so the music generation model based on music theory rules extracts the features of real chords for mechanical music generation. The principle of backpropagation (BP) [28, 29] is adopted, as shown in Figure 6:

In Figure 6, backpropagation is divided into forward-propagation and back-propagation. The forward process assumes an *x* is input. Its weight is set to *w*, and the two are multiplied to obtain and then subtracted from the real *y* value to obtain the error valuer. The square of the error value is the loss value of the function, and the forward propagation ends. Then, the loss value is partially differentiated to complete backpropagation, as shown in the following equations:

(6) $$\begin{array}{c} \text{Loss}={\left(\overset{⟶}{y}-y\right)}^{2}={\left(x\cdot w-y\right)}^{2}, \end{array}$$

(7) $$\begin{array}{c} \frac{\partial \text{Loss}}{\partial w}=\frac{\partial \text{Loss}}{\partial \overset{⟶}{y}}\cdot \frac{\partial \overset{⟶}{y}}{\partial v}= \end{array}$$

The music generation model based on music theory includes three parts: regulator, generator, and discriminator CNNs.  Figure 7 illustrates the structure of the model.

In Figure 7, the input of the regulator CNN in this model is the starting bar melody, which goes through four layers of convolution. The features of the starting subsection are extracted from each layer and are concatenated with the corresponding transposed convolutional layer in the generator. The input of the discriminator CNN is the real melody, or the generated melody goes through two convolutional layers and one fully connected layer to identify the input melody. The discriminator's discrimination performance is continuously improved after rounds of training.

#### 3.4.3. GAN Music Generation Model Based on Chord Characteristics

The structure of the deep chord convolutional generative adversarial network (DCC_GAN), a GAN network music generation model based on chord features, is shown in Figure 8:

In Figure 8, the GAN music generation model based on chord features adds chord CNN to the music generation model based on music theory features. It contains four parts regulator, generator, discriminator, and polyphonic CNN. The generated melody can learn the melody features at time *t* − 1, which has more contextual coherence and fluency.

In the DCC_GAN model, the input of the regulator CNN is the two-dimensional conditional matrix of the note number *h* and the time step *w*. After four layers of convolution, the convolution of each layer is processed by normalization. In equation (8), it can improve the stability of the model and avoid the collapse of the network performance when the input data are too large.

(8) $$\begin{array}{c} y=\frac{x-\text{mean}\left(x\right)}{\sqrt{\text{Var}\left(x\right)}+eps}*\text{gamma}+\text{beta,} \end{array}$$

where *eps* is a constant, the number of columns of melody *x* is input. gamma and beta are parameters of the coefficient matrix. The calculation results are integrated through Leaky ReLU activation function. In equation (9), *a*_*i*_ represents different coefficients and *i* denotes different channels, if *x*_*i*_ > 0 and remains linear, when *x*_*i*_ > 0, data are integrated according to parameters.

(9) $$\begin{array}{c} \text{LReLU}\left(x_{i}\right)=\left\{\begin{array}{cc} x_{i}, & \text{if}x_{i}>0,\\ a_{i}x_{i}, & \text{if}x_{i}\leq 0. \end{array}\right) \end{array}$$

The generator inputs random noise with length *l* = 100 and one-dimensional conditional chord. The composition of chord is to add the conditional vector with length *n* to the middle layer with shape *a∗b*, repeat *a∗b* times, and finally generate the tensor with shape *a∗b∗n*. The tensor of this one-dimensional condition is used as the input of the generator together with Gaussian noise. It passes through dropout layer [30] to prevent over fitting and improve the generalization ability of the model, and then passes through a full connection layer to make the number of neurons reach 1024. The model has undergone four times of transpose convolution, and each time it is normalized and processed by activation function, so that the corresponding nonlinear transformation can be fitted. Chord features will be added in the transposed volume set of each layer to make the generated melody more stable and harmonious. Additionally, each layer will be spliced with the regulator CNN to make the generated melody learn with the starting section as a priori knowledge, increase the interest of the generated melody, and finally generate a two-dimensional piano roll format picture.

The input of the discriminator is the real melody *X* or the generated melody *G*(*z*), and the variables are mapped between (0, 1) through the sigmoid function to achieve the effect of secondary classification, identify whether the incoming melody belongs to the real melody or the generated melody, and feedback the results to the generator CNN, to improve the ability of the generator to generate melody.

Chord CNN consists of four parts: chord feature extraction, chord coding, chord prediction, and chord context correlation. In the calculation process, the melody is mainly transmitted in the form of piano roll, and the original chord is converted to form a tensor with matching shape. The chord features are extracted by splicing the original generator CNN.

#### 3.4.4. GAN Music Generation Model Based on Overall Style

The GAN network music generation model, deep chord gated recurrent neural generative adversarial network (DCG_GAN), is based on the overall style, as shown in Figure 9:

In Figure 9, the overall style-based GAN network music generation model replaces the chord CNN module with the gated recurrent unit (GRU) [31, 32] module. The model consists of four parts: regulator CNN, generator CNN, discriminator CNN, and chord GRU. The purpose is that the model can autonomously learn the chord at time 1: *t* − 1 and generate the chord at time *t*. By preserving the hidden layer state of each batch, the GRU of one layer is constructed and combined with the generator to achieve the effect of automatically learning the overall style of the chord. This model can strengthen the contextual association between the generated musical phrase samples and can also increase the repetition of musical passages, optimize the pleasantness of the generated musical samples, strengthen the deep association between independent samples, and optimize the transition and connection of notes.

GRU is a kind of RNN to achieve the effect of learning the overall style of music [33]. The chord GRU module is to save the hidden state of each batch during the training process. After one round of training, the parameters are sent to the GRU. The constructed 1-layer GRU is transposed and convoluted with the generator, respectively. Chords through GRU generate new chords through the chord coding module, chord prediction module, and chord context-related module and send them to the next round of input. In this way, the model can independently learn the chord content at time 1, *T* − 1, automatically generate the chord at time *t*, automatically learn the overall style of the chord, and then affect the generated content of the whole melody.

### 3.5. Music Generation Experiment and Evaluation

The music generation model, DCC_GAN, and DCG_GAN model based on music theory knowledge generate a huge number of musical melodies. Compared with the baseline model Midinet, the generated melodies are more coherent and pleasant. The generated music is iterated for different rounds (1 epoch, 100 epoch, and 200 epoch) to get the generated melody. There is no rigorous, objective evaluation standard for the evaluation of music. The ultimate purpose of music is for people to enjoy, so people's subjective evaluation is also very important. A music evaluation method based on subjective evaluation and objective indicators is designed to verify the effectiveness of the model improvement scheme.

The subjective evaluation adopts the method of an online questionnaire survey of volunteers and uses the Internet platform to conduct the anonymous evaluation. The melodies generated by the baseline model, the music generation model, the DCC_GAN model, and the DCG_GAN model are numbered. Volunteers can only see the number without knowing other music information, which allows the evaluation to exclude other interference, and the results are more objective. Differences in volunteers' cognitive levels of music impact the structure. Therefore, volunteers are divided into professional musicians and ordinary listeners according to their professional background in music. Those who have systematically learned the knowledge of music theory or mastered any musical instrument are positioned as professional musicians, and the rest are ordinary listeners. In the end, ten professional musicians are selected, and 40 general listeners are tested. In the questionnaire, three subjective evaluation indicators are set, namely the contextual coherence between the musical sample phrases, the musicality of the phrases, and the authenticity of the musical sample. A scoring system of 1–5 is adopted, taking coherence as an example, with five being very coherent, one being very incoherent, and so on.

Then, the above evaluation results are further analyzed. The results of the GAN dual-track music generation model based on chord constraints are weighted and averaged. The score of ordinary listeners is calculated according to the ratio of 40%, and the score of professional musicians is calculated according to 60%, as shown in the following equation :

(10) $$\begin{array}{c} \bar{x}=\frac{x_{1}f_{1}+x_{2}f_{2}+x_{3}f_{3}+\cdots x_{k}f_{k}}{\sum_{1}^{k}f_{i}}. \end{array}$$

The weights of context coherence, phrase rhythm, and pleasantness among music sample phrases and the authenticity of music samples are analyzed according to 5 : 3:2, and the evaluation results are obtained.

In addition, rhythm and pleasantness are the core of the three evaluation criteria, and the correlation with the other two evaluation criteria needs to be analyzed. The Pearson correlation coefficient is used to evaluate, as shown in the following equation:

(11) $$\begin{array}{c} r=\frac{N\sum x_{i}y_{i}-\sum x_{i}y_{i}}{\sqrt{N{\sum x_{i}}^{2}-{\sum x_{i}}^{2}\sqrt{N{\sum y_{i}}^{2}-{\sum y_{i}}^{2}}}}. \end{array}$$

The objective evaluation adopts the objective evaluation method proposed by the Muse GAN model based on some characteristics of music data, such as empty bars rate (EBR), UPC, and qualified note ratio (QNR). EBR refers to the ratio of non-note empty bars to the total number of bars generating music samples in track music bars. UPC refers to the number of pitch level types contained in each section of the track of the music sample, ranging from 0 to 12. QNR is the ratio of qualified notes to the number of bar notes in the bar where the music sample is generated. The judgment standard is that when the duration of a note is less than three standard time steps (32-minute notes), it is judged as an unqualified note.

## 4. Results

### 4.1. Melody Generated by Different Music Generation Models

MIDI format music is displayed in the form of piano volume through MIDI Editor software, and the first four sections of each melody are selected, as shown in Figure 10.

In Figure 10, both the melody and chord generation results of the baseline model Midinet tend to be flat; the melody part of the generation model based on music theory rules is richer; DCC_GAN chords and melody changes are more abundant, but the chords in the middle two bars are still connected. The experimental results of the DCG_GAN model have large changes in both chords and melody, and the melody is more constrained by chords, making the generated music more coherent.

### 4.2. Subjective Evaluation Results of Listeners with Different Music Generation Models

The subjective evaluation adopts the method of an online questionnaire survey of volunteers and uses the Internet platform to conduct the anonymous evaluation. The melodies generated by the baseline model, the music generation model, the DCC_GAN model, and the DCG_GAN model are numbered. Volunteers can only see the number and no other music information. The evaluation results of volunteers scoring different music generation models are shown in Figure 11:

In Figure 11, the overall style-based GAN network music generation model DCG_GAN has the highest score among the four models in terms of music context coherence, pleasantness, and authenticity score, reaching 3.8 points. Compared with the baseline model, the biggest difference in scores is the evaluation of professional musicians in the direction of coherence, and DCG_GAN is 1.4 points higher. The smallest difference in ratings is the rating of ordinary listeners in the direction of authenticity, with a difference of only 0.4 points. It shows that the user's discrimination between the generated music and the real music is not obvious, which further shows the superiority of the DCG_GAN generation model.

Figure 12 presents the scoring results obtained after the weighted average of different generation models.

In Figure 12, the model performance is gradually improved, and the generated music melodies are more realistic and pleasing to the ear. The scores of the three evaluation indicators of DCG_GAN are all the highest. The average score given by ordinary listeners reaches 3.76 points, and the professional score reaches 3.58 points, which are 0.69 and 1.31 points higher than the baseline model, respectively. Therefore, the music generation model based on chord constraints and overall style has more superior performance.

Figure 13 suggests the correlation analysis between the musical melody rhythm and sweetness of different generation models and the other two evaluation criteria.

In Figure 13, the correlation coefficients between the musical melody rhythm and pleasantness and between the phrase rhythm, pleasantness, and the authenticity of the music samples of different models are at least 0.385, all showing a positive correlation.

### 4.3. Audience Objective Evaluation Results of Different Music Generation Models

The evaluation results of the objective evaluation indexes EBR, UPC, and QNR of the four music generation models are shown in Figure 14:

In Figure 14, the first column of the histogram represents the quantized values of the training data, and the remaining columns represent the quantized values of different music generation models. The performance of music sample data generated by the overall style-based DCG_GAN model is closer to the real music training data set on these objective metrics. In the EBR, the music samples generated by the DCG_GAN model have a higher ratio of empty bars and generated music samples in the bass and guitar tracks without notes. Based on music theory, the gaps between DCC_GAN and DCG_GAN and the baseline model are 25.789%, 23.56%, and 15.485%, respectively. DCG_GAN is 8.075% better than DCC_GAN.

In the UPC evaluation data, except for the piano track, the DCG_GAN model performs better than the DCC_GAN model based on music theory, and the most improved is in the guitar track. The DCG_GAN model outperforms the baseline model by 0.52.

In the QNR evaluation index, the DCG_GAN model has different degrees of improvement in the five audio tracks than the DCC_GAN model, up to 4.46%. The overall performance of the improved DCG_GAN music generation model based on the overall style is the best, and the generated notes are closer to the real melody.

## 5. Conclusion

Music, as a carrier of human expression of emotion, has achieved rapid progress in music creation combined with modern information technology. Through the study of music generation methods and music creation psychology, the important role of chords in music expression is introduced, and the CNN-based baseline model Midinet is proposed. A GAN music generation model based on music theory rules and chord features and based on overall style is constructed. The generated melodies are compared in a comprehensive evaluation of subjective and objective directions. The results show that the music generated based on chord constraints is closer to the real melody, which provides a basis for psychological education research on music creation. However, some deficiencies still exist. Although the generated music melodies have been optimized, the generation model is based on dual track-generated melodies. In the future, the generation effect of the model in multi-track music will be further added with different instruments to generate richer melodies.

## Figures and Tables

**Figure 1:** Schematic diagram of MIDI file parsing process.

**Figure 2:** The structure of GAN.

**Figure 3:** Structure of Midinet model.

**Figure 4:** Structure of discriminator and generator network ((a) discriminator network and (b) generator network).

**Figure 5:** The preprocessing process of the music generation data set.

**Figure 6:** The principle of backpropagation.

**Figure 7:** Music generation model based on music theory rules.

**Figure 8:** GAN music generation model based on chord characteristics.

**Figure 9:** GAN music generation model based on overall style.

**Figure 10:** Experimental results of different music generation models ((a) baseline model, (b) based on music theory, (c) DCC_GAN, and (d) DCG_GAN).

**Figure 11:** Experimental subjective evaluation results of different music generation models ((a) the scores of ordinary listeners and (b) the scores of professional musicians).

**Figure 12:** Melody-weighted average results generated by four groups of models.

**Figure 13:** Correlation analysis between evaluation criteria of different models.

**Figure 14:** Comparison of objective evaluation index results of different models: (a) comparison of the ratio of empty bars without notes in different models to the total number of bars of generated music samples; (b) comparison of the number of pitch grade types contained in different models; and (c) comparison of the ratio of qualified notes in bars of different models.

**Table 1:** Compilation environment settings of music generation model.

Name	Settings	Advantages/effects
Operating system	Linux operating system	Stable, free, multitask and multi-user operation, low internal consumption, etc
Network implementation framework	Pytorch network framework	Dynamic calculation diagram, easy to understand code, GPU acceleration, and high model learning efficiency

Main Python libraries	Pypianoroll	MIDI files can be parsed into multi-track piano volumes, and multi-track piano volumes can also be compiled into MIDI files to realize the mutual conversion between piano volumes and MIDI files.
	Xml.Etree.Element Tree	Get data set
	Xml dataset	Tag data set
	Mat	Provide common mathematical operations
	Matplotlib	Drawing tools
	Numpy	Realize the operation of array and matrix of advanced dimensions
	ipdb	Debug Python code command line

## Data Availability

The simulation experiment data used to support the findings of this study are available from the corresponding author upon request.
